# Safety and Efficacy of CT-Guided Central Venous Catheter Gastric Insufflation in Percutaneous Gastrostomy

This article has been retracted.

**DOI:** 10.1155/2022/9421738

**Published:** 2022-09-29

**Authors:** Wen Zhang, Ruoyu Deng, Boyu Chen, Jialing Lv, Tingbiao Zhu, Meifang Huang, Guoyu Xu, Feineng Liu, Tengfei Zhang, Lin Wang, Jun Yue, Lixia Mu, Chao Zhang

**Affiliations:** Department of Oncology, The First People's Hospital of Qujing, Qujing 655000, China

## Abstract

Gastric insufflation for computed tomography (CT)-guided percutaneous gastrostomy is currently performed via a nasogastric tube or a Chiba needle. However, nasogastric tube placement requires patient pharynx and esophagus, and Chiba needle use is associated with an increased risk of organ damage and prolonged operation time. Herein, we introduce a new method of gastric insufflation via a central venous catheter and explore its safety and efficacy by retrospective analysis of the clinical data of patients who underwent percutaneous gastrostomy using this method in our hospital from April 2021 to March 2022. The extracted data included the following: success rate, operation time, gastric insufflation time, radiation dose, postoperative pain score, and complications. We also compared the preoperative levels of several nutritional indicators (body mass index, hemoglobin, albumin, creatinine, and blood urea nitrogen) with those obtained 1 month postoperatively. A total of 12 patients underwent percutaneous gastrostomy under CT guidance using central venous catheter gastric insufflation. The surgery and gastric insufflation success rates were 100% both. The average operation time, gastric insufflation time, and effective radiation dose were 24.08 ± 5.25 min, 5.08 ± 2.50 min, and 14.16 ± 3.63 mSv, respectively. Based on the World Health Organization scale for pain assessment, five patients reported no postoperative pain and seven patients had mild pain. There were no serious complications, such as stoma infection, peritonitis, gastrointestinal perforation and bleeding, or embedding syndrome. All evaluated nutritional indicators showed improvement at 1 month postoperatively, with statistically significant differences compared to the preoperative values (*p* < 0.05 for all). In conclusion, CT-guided percutaneous gastrostomy with central venous catheter gastric insufflation is a safe, effective, and feasible minimally invasive treatment.

## 1. Introduction

Computed tomography (CT)-guided percutaneous gastrostomy requires dilation of the stomach to ensure that it is closely adhered to the abdominal wall. Currently, there are two methods of gastric insufflation: via a nasogastric tube and a Chiba needle [1]. However, both these methods have certain disadvantages. Namely, patients with severe esophageal stenosis and occlusion are ineligible for nasogastric tube placement. Furthermore, in a recent study comparing these two methods, despite the lack of differences in the operation success rate, the Chiba needle was found to be inferior to the nasogastric tube because it is relatively hard to use and not easy to bend, which increases the risk of organ damage and prolongs the operation time, resulting in a higher operation cost and radiation dose [2].

Therefore, we explored the feasibility, efficacy, and safety of a new method of gastric insufflation using a central venous catheter (CVC). To the best of our knowledge, no studies have reported the use of CVC gastric insufflation in CT-guided percutaneous gastrostomy.

## 2. Materials and Methods

### 2.1. Study Design and Population

This was a retrospective analysis of the clinical data of patients who underwent CT-guided percutaneous gastrostomy using CVC gastric insufflation in our hospital from April 2021 to March 2022. All patients were ineligible for nasogastric tube placement and were evaluated to be at high risk of malnutrition according to the Nutritional Risk Screening-2002 tool for nutritional risk assessment in hospitalized patients. All patients provided written informed consent for participation in the study.

### 2.2. Equipment

CT guidance was achieved using a 16-row large-bore helical CT simulator (Brilliance CT Big Bore, Philips). A custom-made body surface positioning grid was used to determine the optimal puncture point. A disposable CVC kit (CVC-1, 16G, 20, adult FORNIA) was used for gastric insufflation (Figure 1). The gastrostomy equipment included a gastric wall fixator, a three-way device, and a gastrostomy puncture kit (Tonda-style gastrostomy kit PEG-15, Japan Couliette).

### 2.3. Preoperative Preparation

All patients underwent routine laboratory evaluation, including routine blood tests, liver and kidney function tests, and coagulation tests; four mandatory inspections; and imaging evaluation, including abdominal contrast-enhanced CT, electrocardiography (ECG), cardiac function tests, and upper gastrointestinal CT angiography. Warfarin was discontinued for 3–5 days, low-molecular-weight heparin for 8 h, and antiangiogenic drugs 4–6 weeks preoperatively. Patients were fasting for 8 h before the surgery. Anisodamine (6542) 10 mg was injected intramuscularly for 15 min, and venous access was established. Patients were placed in the supine position on the CT scanning bed, and ECG monitoring was connected.

### 2.4. Surgical Technique

#### 2.4.1. Gastric Insufflation

After the positioning grid was attached to the surface of the upper abdomen parallel to the long axis of the body, CT of the upper abdomen was performed. The optimal puncture point, angle, and depth were determined according to the CT images. The surgical field was routinely disinfected and isolated with compresses, after which local anesthesia was administered using 5 mL of 2% lidocaine at the puncture point and subcutaneous tissue up to the peritoneum. The puncture needle was inserted in accordance with the predetermined puncture point, angle, and depth until there was a sense of loss of resistance. A CT scan was obtained to confirm that the puncture needle tip is located in the stomach (Figure 2). Next, the guide wire was removed from the puncture needle and the CVC was inserted. Another CT scan was obtained to confirm that the catheter is located in the stomach (Figure 3), after which 1,000–1,500 mL of air was slowly injected through the catheter. The amount of gas injected was adjusted based on the size, degree of expansion, and level of adherence of the stomach to the abdominal wall. A CT scan was performed again to ensure that the gastric cavity was fully filled and tightly adhered to the abdominal wall, and a 5 mL syringe needle was used as a reference to determine the location of the gastrostomy puncture point.

#### 2.4.2. Gastric Puncture and Gastric Wall Fixation

After administering local anesthesia (5 mL of 2% lidocaine) at the gastrostomy puncture point and surrounding skin (about 3 cm in diameter), the gastric wall fixator was positioned vertically over the gastric wall, centering on the site of the intended gastrostomy opening and 1 cm laterally, and the needle was inserted until there was a sense of loss of resistance. A CT scan was obtained to confirm that the needle tip of the gastric wall fixator is located in the stomach (Figure 4). The blue needle core was pushed in, the yellow needle core was pulled out, a silk thread was inserted through the yellow coaxial puncture needle, and the blue needle core was lifted until there was a sense of slight resistance. Next, the gastric wall fixator was pulled out, the sutures of the two needles were guided to the external ligation, and the gastric and abdominal walls were symmetrically ligated and fixed with the predetermined gastrostomy opening as the center (Figures 4 and 5).

#### 2.4.3. Insertion and Fixation of the Gastrostomy Tube

The PS needle with a T-shaped peelable sheath was inserted into the stomach vertically through the predetermined puncture point (Figure 6). The peelable sheath was pushed, and a CT scan was performed to confirm that the tip of the peelable introducer sheath was located in the gastric cavity. The needle was removed, the air outlet was blocked with fingers, the gastrostomy tube was quickly inserted into the gastric cavity through the peelable introducer sheath, and 5 mL of sterile water for injection was injected through the water injection port to fill the tube tip balloon. After confirming that the gastrostomy tube is located in the stomach, the T-shaped sheath was peeled off and removed, and the gastrostomy tube was pulled outward to ensure adherence of the anterior stomach wall with the abdominal wall. The stoma plate was pressed against the abdominal wall to ensure fixation, the gas from the stomach was removed, and 200 mL of diluted contrast medium was injected through the gastrostomy tube to check the patency of the stoma (Figures 7 and 8). After confirming absence of contrast leakage, the surgery was ended.

### 2.5. Postoperative Care

Regular ECG and vital sign monitoring was performed 24 h after the surgery. Patients were closely monitored for any complications. Stoma care included cleaning of the skin around the fixed plate, daily dressing change for 1 week after the surgery, and timely intervention in case of redness and swelling of the wound. After initial warm saline boluses, patients were gradually transitioned to a liquid diet. The tube was cleaned with warm boiled water before and after each injection to prevent the tube from being blocked. If the tube was blocked, it was flushed using a 5 mL syringe, and if necessary, a guide wire was used to clear the tube. To prevent gastrostomy tube prolapse, the saline solution in the balloon was replaced every 3–5 days.

### 2.6. Follow-Up

Patients were reevaluated 1 month after the surgery to determine the stoma and gastrostomy tube status, check for any complications, and measure the level of the nutritional indicators (body mass index, hemoglobin, albumin, creatinine, and blood urea nitrogen). The survival status was recorded by telephone or outpatient follow-up for more than 3 months.

### 2.7. Statistical Analysis

IBM SPSS Statistics version 25.0 (IBM Corp., Armonk, NY, USA) was used for statistical analysis. Measurement data were expressed as mean ± standard deviation (*x* ± *s*) and compared using the paired *t*-test. Enumeration data were expressed as cases or percentages (%). A *p*-value less than 0.05 was considered to indicate statistical significance.

## 3. Results

### 3.1. Patient Characteristics

A total of 12 patients (eight men and four women) with an average age of 59.8 ± 10.4 years (range, 45–76 years) underwent CT-guided percutaneous gastrostomy with CVC gastric insufflation. Among them, six patients had nasopharyngeal cancer, four had esophageal cancer, and two had lung cancer with esophageal stricture. According to the Nutritional Risk Screening-2002 scores, eight patients were at risk of severe malnutrition and four patients were at risk of moderate malnutrition. All 12 patients were deemed ineligible for surgical resection and stent implantation after surgical evaluation.

### 3.2. Operative Status

The surgery was successfully completed in all 12 patients (surgery success rate, 100%). CVC gastric insufflation and gastrostomy tube placement were successfully completed in the initial attempt in all patients. The average operation time was 24.08 ± 5.25 min (Table 1), the average gastric insufflation time was 5.08 ± 2.50 min (Table 2), and the average effective radiation dose was 14.16 ± 3.63 mSv. There were no cases of intraoperative mortality.

### 3.3. Postoperative Status

According to the World Health Organization scale for pain assessment, five patients reported no postoperative pain and seven patients had mild pain; there were no patients with severe pain. After active analgesic treatment, dressing change, tube flushing, and other treatments, the pain gradually subsided. There were no serious complications, such as stoma infection, peritonitis, gastrointestinal perforation and bleeding, or embedding syndrome in any of the patients after the surgery. Gastrostomy tube prolapse occurred in one patient, but the tube was successfully replaced and remained in place thereafter.

### 3.4. Follow-Up

At 1 month postoperatively, all evaluated nutritional indicators were improved, with a statistically significant difference compared to the preoperative values (*p* < 0.05 for all; Table 3). One patient died of tumor rupture 2 months after the surgery, and four patients died of respiratory failure 3 months after the surgery. No gastrostomy-related mortality was recorded.

## 4. Discussion

In this study, we introduced CVC gastric insufflation in CT-guided percutaneous gastrostomy and demonstrated that it is a safe and effective new method that can be applied in patients undergoing this procedure.

Percutaneous gastrostomy can improve the nutritional status and quality of life of patients who cannot feed orally due to pharyngeal or esophageal stenosis [3, 4]. It is a safe and effective enteral nutrition method, particularly useful in patients with advanced-stage pharyngeal and esophageal malignant tumors [5]. The advantages and disadvantages of different guidance methods have always been a research hotspot, but there is little research on the effect of gastric gas injection. Gastric dilation is an indispensable step in percutaneous gastrostomy because good gastric dilation is a prerequisite for the success of the procedure. Optimal gastric dilation provides sufficient gastric wall tension, facilitates the entry of the puncture needle, and can push the surrounding organs to make the stomach wall close to the abdominal wall, which facilitates finding a safer, more direct path into the stomach and avoiding organ damage [6, 7].

Current methods of gastric dilation include gas insufflation using a nasogastric tube or a Chiba needle [8]. While nasogastric tube gas injection is a noninvasive procedure, it is not suitable for all patients, such as those with severe esophageal and pharyngeal strictures, obstructions, and gastric position variation; patients who cannot pass gastric tubes; and those who refuse gastric tube placement. Spelsberg et al. [9] initially investigated the feasibility of gastric insufflation by puncturing the stomach wall with a Chiba needle and achieved good results. Jiang et al. [1] also confirmed that it is feasible to inject gas with a Chiba needle without placing a nasogastric tube. However, a recent study demonstrated that gas injection through a Chiba needle has several drawbacks [2]. First, the Chiba needle has a small diameter and the gas injection speed is slow, which prolongs the operation time. Second, the Chiba needle has a certain hardness and requires more time for placement in the gastric cavity, considering the compression and deformation of the stomach during the operation under the influence of gastric peristalsis and breathing motion, greatly increasing the risk of gastric wall damage. Furthermore, if repeated gas injections are required, the Chiba needle needs to be pulled and inserted repeatedly. The needle core is not only cumbersome to operate but also more likely to cause displacement of the needle tube and air leakage through the needle core. Finally, in patients whose liver or intestinal tract covers the body of the stomach, it is necessary to directly puncture the overlying organs to reach the stomach cavity, which increases the risk of organ damage.

Considering all above, our team explored a new method of gastric insufflation using a disposable CVC. To the best of our knowledge, no studies have reported the use of CVC gastric insufflation in CT-guided percutaneous gastrostomy. CVCs are widely used in clinical practice because of their simple and convenient operation, easy mastering, and high accessibility. They are often used for drug infusion, parenteral nutrition, blood purification, and central venous pressure measurement [10]. In recent years, CVCs have also been applied for drainage of fluid and gas in cases of pericardial and pleural effusion and pneumothorax, with good results [11]. In this study, it was used for the first time to inject gas into the stomach. The advantages of this new method are as follows. First, the technique is simple, the CVC is easy to operate, and the one-time puncture enables repeated gas injection. Second, the CVC has a movable clamping valve, which can be opened and closed at any time according to the needs for gas injection. The possibility of closing the catheter is convenient, as it prevents air leakage and has high reliability. Third, the CVC is mainly made of silicone, which provides better tissue compatibility compared to traditional catheters, greatly reducing infection rates, and softer structure, reducing the probability of organ damage [12]. Finally, the CVC diameter is larger than that of the Chiba needle (16 G vs. 22 G), enabling fast gas injection and deflation and high efficiency.

In this study, CVC placement and gastric dilation were completed successfully in the first attempt in all 12 patients, and the operation success rate was 100%. In the study of Zhao et al. [2], the duration of gastrostomy via the nasogastric tube and that via the Chiba needle was 36.56 ± 6.84 min and 47.17 ± 5.12 min, respectively. Other studies [13] reported a gastrostomy operation time of 45 ± 15 min. In this study, the average operation time was 24.08 ± 5.25 min, with operation completion within 30 min in 83.3% of the patients, and the average gastric insufflation time was 5.08 ± 2.50 min, with procedure completion within 5 min in 66.7% of the patients. Therefore, the use of CVC gas injection for gastrostomy may shorten the operation time. In terms of the effective radiation dose, Spelsberg et al. [9] reported an average effective radiation dose of 7 ± 5.4 mSv in 101 patients who underwent CT-guided gastrostomy. In the study of Zhao et al. [2], the effective radiation doses when using a nasogastric tube and a Chiba needle were 13.95 ± 3.04 mSv and 23.13 ± 5.22 mSv, respectively. The average effective radiation dose in our study was 14.16 ± 3.63 mSv, indicating that CVC gastric insufflation did not significantly increase the radiation dose. However, due to the difference in CT parameters across medical centers, these findings should be verified through further studies.

The comparison of the nutritional indicators (body mass index, hemoglobin, albumin, creatinine, and blood urea nitrogen) between before and 1 month after surgery indicated that the patients' nutritional status was significantly improved. Postoperative pain was the most common complication in this study reported by seven of the 12 patients but was rated as mild and was well controlled with observation or appropriate treatment. The remaining five patients reported no pain. There were no serious postoperative complications in any of the patients or gastrostomy-related mortality during follow-up. Furthermore, it should be noted that the cost of the CVC kit in our hospital is lower than that of the Chiba needle kit, suggesting that this new method can also reduce the cost of surgery.

There are also limitations to this study. First, due to the limited conditions, it was designed as a single-arm study without controls. Second, it was a retrospective analysis and the total sample size was relatively small. Future prospective studies with a larger sample size are warranted to confirm our findings.

## 5. Conclusions

CVC gastric insufflation is a safe and effective method that can reduce the economic burden of patients and provide a new solution for gastric dilation in CT-guided gastrostomy, which supports its clinical application.

## Figures and Tables

**Figure 1:** Disposable central venous catheter kit.

**Figure 2:** Axial computed tomography scan showing that the puncture needle tip is located in the stomach.

**Figure 3:** Axial computed tomography scan showing that the central venous catheter is located in the stomach.

**Figure 4:** Sagittal computed tomography scan showing that the tip of the gastric wall fixator is located in the stomach.

**Figure 5:** Intraoperative image showing that the gastric and abdominal walls were symmetrically ligated and fixed with the gastrostomy opening as the center.

**Figure 6:** Intraoperative image showing the positioning of the PS needle with a T-shaped peelable sheath. The needle was vertically pierced into the stomach through the predetermined puncture point.

**Figure 7:** Axial computed tomography scan showing that the gastrostomy tube tip was placed into the stomach and fixed with the water balloon. No contrast medium extravasation was seen.

**Figure 8:** Postoperative image showing that the stoma fixation plate properly secures the gastrostomy tube to the abdominal wall.

**Table 1:** Computed tomography-guided percutaneous gastrostomy operation time (*n* = 12).

Operation time	*n*	%
10–20 min	4	33.3
21–30 min	6	50.0
>30 min	2	16.7

**Table 2:** Computed tomography-guided percutaneous gastrostomy gastric insufflation time (*n* = 12).

Gastric insufflation time	*n*	%
0–5 min	8	66.7
5–10 min	3	25.0
>10 min	1	8.3

**Table 3:** Comparison of nutritional indicators before surgery and 1 month after surgery (*x* ± *s*).

Grouping	BMI (kg/m^2^)	Albumin (g/L)	Hemoglobin (g/L)	Creatinine (*μ*mol/L)	Urea nitrogen (mmol/L)
Preop	16.74 ± 1.73	29.50 ± 3.89	105.50 ± 17.56	54.75 ± 13.36	3.05 ± 0.94
1 month postop	17.02 ± 1.71	32.83 ± 2.73	110.50 ± 13.50	58.17 ± 11.40	3.74 ± 0.67
*t*	−3.000	−2.626	−2.481	−2.403	−2.316
*p*-value	0.012	0.024	0.031	0.035	0.041

## Data Availability

The data used to support the findings of this study are included within the article.
